# Performance Prediction of Listed Companies in Smart Healthcare Industry: Based on Machine Learning Algorithms

**DOI:** 10.1155/2022/8091383

**Published:** 2022-01-07

**Authors:** Baobao Dong, Xiangming Wang, Qi Cao

**Affiliations:** School of Management, Jilin University, Changchun 130025, Jilin, China

## Abstract

With the development of wireless network, communication technology, cloud platform, and Internet of Things (IOT), new technologies are gradually applied to the smart healthcare industry. The COVID-19 outbreak has brought more attention to the development of the emerging industry of smart healthcare. However, the development of this industry is restricted by factors such as long construction cycle, large investment in the early stage, and lagging return, and the listed companies also face the problem of financing difficulties. In this study, machine learning algorithm is used to predict performance, which can not only deal with a large amount of data and characteristic variables but also analyse different types of variables and predict their classification, increasing the stability and accuracy of the model and helping to solve the problem of poor performance prediction in the past. After analysing the sample data from 53 listed companies in smart healthcare industry, we argued that the conclusion of this study can not only provide reference for listed companies in smart healthcare industry to formulate their own strategies but also provide shareholders with strategies to avoid risks and help the development of this emerging industry.

## 1. Introduction

The World Health Organization defines smart health (eHealth) as the use of information and communication technologies (ICT) to provide comprehensive services in healthcare. The healthcare information system can be more easily managed by improving the design of information flow. This new healthcare mode provides a new path for the development of global healthcare industry. Moreover, with the advent of the aging era, how to live healthy is one of the important issues that modern people pay attention to. Through the application of wireless network communication technology, cloud platform, and Internet of Things (IOT) in healthcare treatment, smart healthcare care has become an indispensable smart health technology for people [1, 2]. In the era of big data, smart healthcare technology can also help improve healthcare efficiency and service quality. More importantly, since the end of 2019, the outbreak of COVID-19 has aroused the importance of Internet healthcare, and the smart healthcare industry has ushered in significant development opportunities, but at the same time, it is also facing great challenges and risks [3]. In order to develop the emerging industry of smart healthcare, sufficient funding is needed. The construction cycle of smart healthcare treatment is long, the initial investment is huge, and the return lags behind [1]. In order not to let the capital chain restrict the development of companies, many smart healthcare companies choose to go public, but the performance of these companies in the stock market is not satisfactory. Many smart healthcare companies are facing serious financial risks and heavy costs, which affect their performance [4–6].

After analysing of the performance of listed companies in the smart healthcare industry, we finds that there are also many problems in the development process of the companies, and the financial risks in its development are relatively large. As an emerging industry, healthcare industry must solve many problems we will face in the future. So, we should give support to this industry. But the current situation is not so amiable to the development of this industry. The development of many companies presents strong fluctuation and instability. Therefore, a detailed analysis of the performance of listed smart healthcare companies can provide valuable reference for the long-term development of companies and shareholders` investment.

However, the current predictive analysis of performance is lack of reasonable explanation, and the research methods are mainly focused on the traditional regression analysis technology to analyse the main influencing factors of performance [7]. For example, Booth, regressed and based on the sample data of 10 countries in developing countries, found that debt service ratio had the same influence on the development of listed companies in both developing and developed countries. The most important factor was profitability, and capital structure had a negative correlation with corporate business performance [8]. Li et al. empirically examined the effect of firm performance on CSR disclosure in terms of disclosure frequency and quality among Chinese listed firms and the possible mediating effect of corporate ownership on the relationship between firm performance and CSR disclosure. They argued that performance influenced CSR and then the future investment [9]. Traditional measurement indicators are based on the assumption of normal distribution, but in fact, the performance of listed smart healthcare companies is not normal distribution, which results in bad prediction of the performance. In this study, machine learning is used to predict performance, which can not only deal with a large amount of data and characteristic variables but also analyse different types of variables and predict their classification, increasing the stability and accuracy of the model and helping to solve the problem of poor performance prediction in the past. This study may be the pioneer to study performance prediction of listed companies in healthcare industry by using machine learning, which can give some hints or directions for future research in prediction for companies.

Therefore, this paper will study the performance of listed companies in the smart healthcare industry, provide reference for companies to formulate their own strategies, and provide shareholders with risk-avoiding strategies to facilitate the development of this emerging industry.

## 2. Literature Review

### 2.1. Operating Performance of Listed Companies

Performance is the result of the enterprise's work to achieve the established goal. Performance of an enterprise refers to the operating results of an enterprise and the performance of an operator during a certain operating period. The level of business efficiency is mainly reflected in the profitability, asset operation level, debt paying ability, and follow-up development ability of the enterprise. The performance of managers is mainly reflected by the achievements and contributions made by managers to the operation, growth, and development of companies in the process of operating and managing companies [1]. Enterprise management performance evaluation includes two aspects of enterprise management benefit and operator performance evaluation.

Listed companies in different industries have different market structure, growth capacity, correlation with macroeconomic cycle, and life cycle stage of the industry, so their business performance is also significantly different. This paper intends to make a comprehensive evaluation of the business performance of listed smart healthcare companies by analysing the index system reflecting the business performance of listed companies in the smart healthcare industry and using the machine learning method. On this basis, it attempts to study the business performance of listed smart healthcare companies in China from the perspective of the industry, so as to provide predictive reference for their future development.

### 2.2. Smart Healthcare Industry

In addition to the definition of eHealth by WHO, some scholars believe that eHealth is also related to public health and commercial healthcare information [7]. Broadly speaking, apart from the technical level, smart healthcare also includes an attitude of thinking to enhance healthcare care [10]. eHealth covers a wide range, including mHealth and smart health [11]. According to the U.S. Food and Drug Administration (FDA), smart healthcare in the broad sense includes mobile healthcare (mHealth), health information technology, wearable devices, remote healthcare, and personalized healthcare technology [12]. Smart healthcare promises to improve overall healthcare efficiency and make it easier for patients and users to track and manage personal health information.

The development of smart healthcare mainly relies on three aspects to build the health data ecosystem. The first is the data source, that is, sensors, wearable devices, and real-time monitoring devices are used to obtain users' physiological health data, and the second is that the above data are combined with more diversified living environment and user behaviour information. The third is to adapt to the technological or industrial environment changes of the first two, and the participation of stakeholders will also change the overall health information environment system [3].

Smart healthcare treatment integrates artificial intelligence, big data, Internet of Things, and other technologies and uses the Internet and other emerging things to integrate resources [12]. Doctors in large hospitals can make inquiries through the computer screen, and the examination data of each hospital can be connected to reduce multiple examinations of patients, and timely investigation of the past healthcare history of patients or emergency patients can greatly facilitate the basic needs of the people, so that doctors can stay at home, and data sharing does not waste healthcare resources. Smart healthcare consists of smart hospital system, regional health system, and family health system.

### 2.3. Machine Learning

Machine learning is a popular algorithm in recent years. In the past, the variables analysed by traditional methods must be independent, and the amount of data should not be too large, especially when extreme values are encountered, which also leads to relatively limited performance prediction [13]. However, machine learning overcomes the limitations of traditional data and adapts to the requirements of the era of big data. It can deal with high-dimensional and nonlinear problems and can not only analyse numerical variables but also explore category-based variables to increase the diversity of variables. The accuracy of prediction is greatly improved by constantly updating the model through learning.

Some scholars have predicted the performance model based on the relevant data of listed companies, which provides valuable reference for the development of listed companies. For example, fund performance can be predicted by multiple fund rating indicators, and fund level can be predicted by random forest, which can not only process high-dimensional data but also perform very well in noise reduction, increasing model stability and improving accuracy. Some scholars studied the time series of financial commodities [14]. Support vector machine (SVM) and random forest can realize the principle of minimum risk, reduce the error ratio, and improve the accuracy of the overall model, which is superior to the general traditional model and neural network analysis methods. Zhang et al. proposed extreme gradient boosting (shortly XGB), which is highly efficient in machine learning algorithm [15]. The above analysis shows that the machine learning algorithm has high precision and reliability for the prediction model of some indicators of listed companies.

## 3. Methodology

### 3.1. Data Collection

The samples in this paper are from listed companies in the smart healthcare industry of the A share of Shanghai and Shenzhen Stock Markets. The sample data are collected from 2015 to 2020. The source of the original data is mainly collected through the Chinese stock market research database developed and produced by Shenzhen Guotai'an Information Technology Co., Ltd. In order to avoid unnecessary errors and the authenticity of the results, the data should be processed as follows:

1. Companies that are not listed within three years are excluded, that is, companies listed after 2017 (including 2017) are not included in the statistical data. Because of their short listing time and insufficient financial data, it is easy to cause sample error.
2. Eliminate ST and ∗ST companies. These companies are generally due to the lack of financial motivation caused by poor management. These companies have extreme performance phenomenon.
3. Eliminate companies with incomplete data in the dataset. Incomplete data may occur during data collection, which may affect the objectivity and impartiality of the results.

Referring to the existing evaluation system at home and abroad, this paper selected sales profit margin, return on assets, asset turnover, cost of sales rate, total asset growth rate, inventory turnover rate, and receivables turnover rate from 53 listed smart healthcare companies as the sample data. The calculation process of each original indicator is shown in Table 1.

### 3.2. Modelling

This research mainly uses machine learning and deep learning for modelling. Machine learning includes logistic regression, random forest and gradient boosting. The above methods are all classification of machine learning, while deep learning is multilayer perceptron [16]. However, we only choose random forest, XGB, and deep learning methods because random forest follows standard procedures to solve problems. It divides problems into several parts, solves them separately, and then combines the results to obtain the required answers. XGB is committed to pushing the lifting tree beyond its computational limits to achieve the engineering goal of fast computation and excellent performance. Deep learning, on the other hand, solves problems in a centralized manner rather than having to break them down [17]. Through the comparison of the two analysis results, we can clearly understand the “interior” of the deep network.

Random forest is a classifier that uses multiple trees to train and predict samples. In machine learning, a random forest is a classifier containing multiple decision trees, and its output categories are determined by the mode of the categories output by individual trees. Leo Breiman and Adele Cutler developed algorithms for random forests. It comes from random decision forests, which were proposed in 1995 by Tin Kam Ho of Bell Laboratories. This approach combines Breimans' “bootstrap aggregating” idea with Ho's “random subspace method” to build a collection of decision trees [18]. It uses the set of trained classifiers to classify new samples and then counts the classification results of all classifiers by majority voting or averaging the output, and the category with the highest result is the final standard [19]. This kind of algorithm can effectively reduce the bias and the number of variation. The random forest flow is shown in Figure 1.

XGB is a general regression analysis algorithm to enhance the performance of basic algorithms. It does not need to construct a high-precision regression analysis, just a rough basic algorithm, and then repeatedly adjust the basic algorithm which can get a better combination of regression model. It can improve the weak learning algorithm to strong learning algorithm and can be applied to other basic regression algorithms, such as linear regression and neural network, to improve the accuracy. Bagging and artificial neural network algorithms are similar but slightly different. The main idea of bagging is to give known weak learning algorithms and training sets. It needs to go through several rounds of calculation to get the prediction function column. The following is the loss function of XGB.

(1) $$\begin{array}{c} L\left(\phi \right)=\sum_{i}l\left({\overset{⌢}{y}}_{i},y_{i}\right)+\sum_{k}\Omega \left(f_{k}\right), \end{array}$$

where *i* represents the *i*th sample, $l\left({\hat{y}}_{i},y_{i}\right)$ represents the prediction error of the *i*th sample, and the smaller the error, the better. ∑_*k*_Ω(*f*_*k*_) is the function of the tree's complexity, the smaller the complexity, the stronger the generalization ability and Ω(f) = *γ*T+1/2*λ*||w||2.

Then, the objective function in iteration *t* can be written as

(2) $$\begin{array}{c} L\left(t\right)=\sum_{i=1}^{n}l\left(y_{i},{\overset{⌢}{y}}_{i}^{t-1}+f_{t}\left(X_{i}\right)+\Omega \left(f_{t}\right)\right). \end{array}$$

Deep learning (DL) is a new research direction in the field of machine learning. It is introduced into machine learning to make it closer to its original goal—artificial intelligence (AI). Deep learning is to learn the internal rules and representation levels of sample data, and the information obtained in the learning process is of great help to the interpretation of data such as text, image, and sound [18, 19].

The concept of deep learning originates from the research of artificial neural network. Multilayer perceptron with multiple hidden layers is a kind of deep learning structure. Deep learning discovers distributed feature representation of data by combining low-level features to form more abstract high-level representation attribute categories or features. The motivation for deep learning research is to build neural networks that mimic the human brain for analytical learning, which can interpret data, such as images, sounds, and texts, by imitating the mechanisms of the human brain [20].

The computation involved in producing an output from an input can be represented by a flow graph: a graph that represents a computation in which each node represents a basic computation and a calculated value, the result of which is applied to the values of the node's children. Consider a set of computations that can be allowed to define a family of functions in each node and possible graph structure.  Figure 2 shows the deep learning model with multiple hidden layers (source: Wei J., Liu A., Tang J., “Alarm model of digital TV monitoring platform: Based on deep learning neural network technology”. *CATV Technology*, vol.11, no.7, pp. 78–82, 2017).

## 4. Performance Evaluation

Random forest, XGB, and deep learning are used to predict the future performance of listed companies in the healthcare industry, that is, whether the performance at next phase will rise or fall, and the confusion matrix is drawn to accurately judge the accuracy, precision, recall, type I error, and type II error [21]. Taking the above five items as the performance evaluation indicators, we will compare the quality of the classification model. Before explaining accuracy, precision, and recall, we need to define the classification of TP, FN, FP, and TN, which are shown in Table 2.

*Accuracy*. The ratio of correctly classified samples to total samples, and it equals to (TP + TN)/(ALL).

*Precision*. Ratio of the number of correctly retrieved samples to total retrieved samples, and it equals to TP/(TP + FP).

*Recall*. Ratio of the number of correctly retrieved samples to the number of samples that should have been retrieved, and it equals to TP/(TP + FN).

The higher the value is, the better the prediction ability is, and the lower it is, the vice versa.

The first type of error, i.e., type I error, refers to the error that rejects H0, which is actually true, and is “truth-rejecting.” Its probability is usually represented by *α*, which is called significance level. *a* can be unilateral or bilateral, generally stipulated *α* = 0.05 or *α* = 0.01.

The second type of error, namely, type II error, refers to the error that does not reject H0, which is actually untenable. It is a “false“ error, and its probability is usually expressed by *ß*. *β* is a single tailed. Generally, the value of *ß* is not known during hypothesis testing, but can be calculated under certain conditions (such as the difference between two populations *δ*, sample content *n*, and test level *α*).  Table 3 shows type I error and type II error.

## 5. Results

In this study, random forest, XGB, and deep learning were used to predict all performance indicators, respectively, in an attempt to compare the accuracy of each machine model in performance prediction. The results are shown in Table 4.

According to the selected important performance variables, machine learning predictions are checked in this study. Table 4 shows that the overall prediction rate of deep learning is the best than that of random forest and XGB. Accuracy, precision, and recall are all higher than those of competitive model. Type I error is also low. However, random forest has a lower type II error. In terms of specific indicators, especially cost of sales rate, the model prediction rate of random forest is the highest than that of deep learning and XGB, but its type I error is higher. In general, deep learning is the best prediction model, while random forest is the best in reducing type II error. In the other six indicators, the predictive power of deep learning has obvious advantages. It can be seen that the deep learning model is more stable for the performance prediction of listed smart healthcare companies.

## 6. Conclusions

In recent years, the number and scale of listed smart healthcare companies are growing steadily. How to acquire stable remuneration among many listed companies has become an important issue. In this study, three kinds of machine learning algorithms are used to predict the future performance of listed companies in the smart healthcare industry. According to the results of accuracy, prediction, recall, type I error, and type II error, deep learning can improve the prediction ability better and stably. There are three findings in this study: first, compared with random forest and XGB, deep learning has relatively stable performance evaluation and accurate prediction, with the lowest type I error. Second, compared with deep learning and XGB, random forest has the lowest type II error. Third, in terms of cost of sales rate, one of the performance indicators, besides type I error, each evaluation index of random forest is better than that of deep learning and XBG. It can be seen that deep learning has the higher accuracy and the prediction model is more stable in predicting the performance of listed companies in smart healthcare industry.

In addition to random forest, XGB, and deep learning, machine learning also includes logistic regression, which also have certain effectiveness for performance prediction. In the future, this model can be applied to the performance prediction model of listed companies to increase the predictive power of the model. In addition, 7 indicators of performance are selected for prediction in this study. In the future, more performance indicators, such as asset-liability ratio, can be added to analyse the development trend of future performance through big data, so as to increase the breadth and accuracy of prediction.

Besides, improving enterprise performance and increasing investor confidence are the main reasons for management to adopt machine learning. These algorithms help enterprise management make correct decisions and mobilize their actions. Machine learning algorithms can provide valuable references for corporate investors to help them avoid risks. Smart healthcare industry is a comprehensive industry integrating health, computer, and artificial intelligence, which has infinite development space in the future. We studied the smart healthcare industry as a whole. So, it is a great pity that it cannot be specific to a specific branch of the smart healthcare industry. In the future, machine learning can be applied to some subindustries of smart healthcare to analyse its future development trend. But no algorithm is optimal, and machine learning is more like an experiment than a Bible.

## Figures and Tables

**Figure 1:** The random forest flow chart.

**Figure 2:** Deep learning model with multiple hidden layers.

**Table 1:** Performance indexes.

Number	Index	Formula	Note
1	Profit margin on sales	Total profit/operation revenue × 100%	It represents the profitability of the enterprise. The higher the index, the stronger the ability of the enterprise to create profits.

2	Return on assets	Net profit after tax/total assets × 100%	It measures how much net profit is generated per unit of assets

3	Asset turnover	Total revenue/total asset × 100%	It measures the efficiency of corporate asset management

4	Cost of sales rate	Sales cost/sales revenue × 100%	It reflects the cost expenditure required by each unit of sales revenue of the enterprise

5	Total asset growth rate	Growth in total assets/total assets at the beginning of the year × 100%	It expresses the capital accumulation ability and development ability of the enterprise

6	Inventory turnover rate	Cost of sales/average inventory × 100%	It reflects the turnover speed of inventory, that is, the liquidity of inventory and whether the amount of inventory capital occupied is reasonable

7	Accounts receivable turnover ratio	Revenue/accounts receivable × 100%	It measures the turnover speed and management efficiency of enterprise accounts receivable

**Table 2:** Confusion matrix.

	Positive	Negative
Retrieved	True positives (TP)	False positives (FP)
Not retrieved	False negatives (FN)	True negatives (TN)

*Note.* TP: positive sample retrieved, actually positive sample (correct identification). FP: positive sample retrieved, actually negative sample (a type of misidentification). FN: positive sample is not retrieved, but is actually positive sample. Type II error identification. TN: the positive sample was not retrieved, which was actually negative sample. (correct identification).

**Table 3:** Type I error and type II error.

	Decision making	
	Accept H0	Reject H0
H0 is true	Correct	Type I error (*α*)
H0 is false	Type II error (*β*)	Correct

**Table 4:** Comparative analysis of performance.

Performance indexes	Evaluation indexes	Random forest	XGB	Deep learning
Profit margin on sales	Accuracy	0.73774	0.70449	0.81584^∗^
	Precision	0.74	0.69	0.83^∗^
	Recall	0.75	0.75	0.80^∗^
	Type I error	0.39176	0.34129	0.28132^∗^
	Type II error	0.09317^∗^	0.17804	0.18359

Return on assets	Accuracy	0.70927	0.73504	0.79304^∗^
	Precision	0.71	0.75	0.80^∗^
	Recall	0.74	0.80	0.83^∗^
	Type I error	0.43914	0.40827	0.30471^∗^
	Type II error	0.08932^∗^	0.12737	0.17588

Asset turnover	Accuracy	0.80931	0.83649	0.84297^∗^
	Precision	0.70	0.77	0.84^∗^
	Recall	0.71	0.74	0.82^∗^
	Type I error	0.38394	0.35127	0.20315^∗^
	Type II error	0.09355^∗^	0.24294	0.16721

Cost of sales rate	Accuracy	0.80319^∗^	0.79339	0.80171
	Precision	0.85^∗^	0.81	0.80
	Recall	0.79^∗^	0.76	0.74
	Type I error	0.43086	0.35149	0.28413^∗^
	Type II error	0.08047^∗^	0.17306	0.14931

Total asset growth rate	Accuracy	0.80106^∗^	0.79254	0.79538
	Precision	0.75	0.77	0.84^∗^
	Recall	0.74	0.73	0.81^∗^
	Type I error	0.50179	0.38147	0.30147^∗^
	Type II error	0.05142^∗^	0.11597	0.10789

Inventory turnover rate	Accuracy	0.78505	0.76582	0.81137^∗^
	Precision	0.80	0.81	0.87^∗^
	Recall	0.79	0.82	0.84^∗^
	Type I error	0.36921	0.30297	0.20762^∗^
	Type II error	0.09399^∗^	0.27446	0.17582

Accounts receivable turnover ratio	Accuracy	0.74209	0.76934	0.81776^∗^
	Precision	0.81	0.80	0.84^∗^
	Recall	0.77	0.79	0.84^∗^
	Type I error	0.46237	0.35887	0.28149^∗^
	Type II error	0.08337^∗^	0.13572	0.14642

^∗^indicates that the value is superior to the competitive model.

## Data Availability

The data used to support this study are available upon request.
